The article "Genetic Polymorphism of Glucokinase on the Risk of Type 2 Diabetes and Impaired Glucose Regulation: Evidence Based on 298, 468 Subjects" was retracted in 2021. Reasons: signs of a paper mill; concerns about the data; concerns about the authorship.

# Genetic Polymorphism of Glucokinase on the Risk of Type 2 Diabetes and Impaired Glucose Regulation: Evidence Based on 298, 468 Subjects

**DOI:** 10.1371/journal.pone.0055727

**Published:** 2013-02-18

**Authors:** Da Fu, Xianling Cong, Yushui Ma, Haidong Cai, Mingxiang Cai, Dan Li, Mingli Lv, Xueyu Yuan, Yinghui Huang, Zhongwei Lv

**Affiliations:** 1 Department of Nuclear Medicine, Shanghai 10th People’s Hospital, Tongji University School of Medicine, Shanghai, People’s Republic of China; 2 China Japan Union Hospital, Jilin University, Changchun, People’s Republic of China; University of Cagliari, Italy

## Abstract

**Background:**

Glucokinase (*GCK*) is the key glucose phosphorylation enzyme which has attracted considerable attention as a candidate gene for type 2 diabetes (T2D) based on its enzyme function as the first rate-limiting step in the glycolysis pathway and regulates glucose-stimulated insulin secretion. In the past decade, the relationship between *GCK* and T2D has been reported in various ethnic groups. To derive a more precise estimation of the relationship and the effect of factors that might modify the risk, we performed this meta-analysis.

**Methods:**

Databases including Pubmed, EMBASE, Web of Science and China National Knowledge Infrastructure (CNKI) were searched to find relevant studies. Odds ratios (ORs) with 95% confidence intervals (CIs) were used to assess the strength of association.

**Results:**

A total of 24 articles involving 88, 229 cases and 210, 239 controls were included. An overall random-effects per-allele OR of 1.06 (95% CI: 1.03–1.09; *P*<10^−4^) was found for the *GCK* −30G>A polymorphism. Significant results were also observed using dominant or recessive genetic models. In the subgroup analyses by ethnicity, significant results were found in Caucasians; whereas no significant associations were found among Asians. In addition, we found that the −30G>A polymorphism is a risk factor associated with increased impaired glucose regulation susceptibility. Besides, −30G>A homozygous was found to be significantly associated with increased fasting plasma glucose level with weighted mean difference (WMD) of 0.15 (95%: 0.05–0.24, *P* = 0.001) compared with G/G genotype.

**Conclusions:**

This meta-analysis demonstrated that the −30G>A polymorphism of *GCK* is a risk factor associated with increased T2D susceptibility, but these associations vary in different ethnic populations.

## Introduction

Type 2 diabetes (T2D) is a complex metabolic disease characterised by hyperglycemia, insulin resistance, impaired insulin secretion due to pancreatic β-cell defects and increased hepatic glucose production. Despite much investigation, the causes underlying the development and progression of T2D have not been fully elucidated, accumulated evidence suggests that multiple genetic and environmental factors, as well as the interplay between these factors, determine the phenotype. Although the genetic contribution to T2D is well recognized, the current set of 56 established susceptibility loci, identified primarily through large-scale genome-wide association studies (GWAS), captures at best 10% of familial aggregation of the disease [1]–[3]. This has maintained interest in other biochemical and genetic factors that might contribute to the underlying pathophysiology of the disease.

The article "Genetic Polymorphism of Glucokinase on the Risk of Type 2 Diabetes and Impaired Glucose Regulation: Evidence Based on 298, 468 Subjects" was retracted in 2021. Reasons: signs of a paper mill; concerns about the data; concerns about the authorship.

Glucokinase (*GCK*) is the key glucose phosphorylation enzyme responsible for the first rate-limiting step in the glycolysis pathway and regulates glucose-stimulated insulin secretion from pancreatic β-cells and glucose metabolism in the liver [4]. Inactivating *GCK* mutations lead to maturity-onset diabetes of the young and neonatal diabetes [5]–[7], whereas activating *GCK* mutations cause persistent hyperinsulinaemic hypoglycaemia [8]–[11]. Moreover, a common variant (−30G>A, rs1799884) in the pancreatic beta cell-specific promoter of *GCK* has been shown to be associated with increased risk of type 2 diabetes, hyperglycaemia and impaired beta cell function [12]–[16]. Furthermore, GCK −30 A>G has been conclusively associated with fasting glucose in European populations [17].

To date, many case–control studies have been carried out to investigate the role of the *GCK* −30G>A polymorphism in the development of T2D among various populations. Genetic association studies can be problematic to reproduce due to insufficient power, multiple hypothesis testing, population stratification, source of controls, publication bias, and phenotypic heterogeneity. In addition, with the increased studies in recent years among Asian, and other populations, there is a need to reconcile these data. We therefore conducted a comprehensive meta-analysis to quantify the overall risk of *GCK* −30G>A polymorphism on developing T2D.

## Materials and Methods

### Literature Search Strategy

Genetic association studies published before the end of Sep. 2012 on T2D and polymorphisms within GCK gene were identified through a search of PubMed, ISI Web of Science, EMBASE and CNKI (Chinese National Knowledge Infrastructure) without language restrictions. Search term combinations were keywords relating to the glucokinase gene (e.g., “glucokinase”, “GCK”, and “MODY 2”) in combination with words related to T2D (e.g., “type 2 diabetes mellitus”, “T2DM”, “type 2 diabetes”, “T2D”, “non-insulin-dependent diabetes mellitus” and “NIDDM”) and polymorphism or variation. The search was supplemented by reviews of reference lists for all relevant studies and review articles. The major inclusion criteria were (a) original papers containing independent data, (b) case–control or cohort studies and (c) genotype distribution information or odds ratio (OR) with its 95% confidence interval (CI) and P-value. The major reasons for exclusion of studies were (a) overlapping data and (b) case-only studies, family-based studies and review articles.

The article "Genetic Polymorphism of Glucokinase on the Risk of Type 2 Diabetes and Impaired Glucose Regulation: Evidence Based on 298, 468 Subjects" was retracted in 2021. Reasons: signs of a paper mill; concerns about the data; concerns about the authorship.

### Data Extraction

Data extraction was performed independently by two reviewers, and differences were resolved by further discussion among all authors. For each included study, the following information was extracted from each report according to a fixed protocol: first author’s surname, publication year, definition and numbers of cases and controls, diagnostic criterion, frequency of genotypes, source of controls, age, gender, body mass index (BMI), Hardy–Weinberg equilibrium status, ethnicity and genotyping method. Not all researchers use the same SNP, we report herein 2 common SNPs (rs1799884 and rs4607517), as these SNPs are in complete disequilibrium (r^2^ = 1) [18].

### Statistical Methods

The strength of association between −30G>A polymorphism of *GCK* and T2D risk was assessed by odds ratio (OR) with the corresponding 95% confidence interval (CI). We first used the chi square test to check if there was significant deviation from Hardy–Weinberg equilibrium among the control subjects in each study. The meta-analysis examined the association between each polymorphism and the risk of T2D for the: (i) allele contrast, (ii) dominant, and (iii) recessive model. For continuity variable, weighted mean difference (WMD) was used to pool results from studies.

Heterogeneity across individual studies was calculated using the Cochran chi-square Q test followed by subsidiary analysis or by random-effects regression models with restricted maximum likelihood estimation [19]–[21]. Random-effects and fixed-effect summary measures were calculated as inverse variance-weighted average of the log OR. The results of random-effects summary were reported in the text because it takes into account the variation between studies. In addition, we investigated potential sources of identified heterogeneity among studies by stratification according to the number of T2D cases (≥1000 and <1000), ethnic group and diagnostic criteria (WHO, ADA or other criterion). Ethnic group was defined as Asians, Caucasians (i.e. people of European origin) and others (e.g. Tunisian and African–American). The Z test was used to determine the significance of the pooled OR. Gender distribution in cases and controls, genotyping method and mean age of cases and controls were analysed as covariates in meta-regression. The transcript expression level trends by genotypes were evaluated by using general linear model.

The article "Genetic Polymorphism of Glucokinase on the Risk of Type 2 Diabetes and Impaired Glucose Regulation: Evidence Based on 298, 468 Subjects" was retracted in 2021. Reasons: signs of a paper mill; concerns about the data; concerns about the authorship.

We assessed publication bias by using an ancillary procedure attributed to Egger et al. [22], which uses a linear regression approach to measure funnel plot asymmetry on the natural logarithm of the OR. Sensitivity analysis was performed by removing each individual study in turn from the total and re-analysing the remainder. This procedure was used to ensure that no individual study was entirely responsible for the combined results. All statistical analyses were carried out with the Stata software version 10.0 (Stata Corporation, College Station, TX, USA). The type I error rate was set at 0.05. All the P-values were for two-sided analysis.

## Results

### Characteristics of Studies

Study selection process was shown in Figure S1. In all, we included 36 data points from 24 studies in this meta-analysis, with a total of 88, 229 cases and 210, 239 controls [12]–[14], [16], [18], [23]–[41]. The distribution of genotypes in the controls was consistent with Hardy–Weinberg equilibrium in all studies. Of the cases, 75% were Caucasians 21% were Asians and 4% were of other ethnic origins. The main study characteristics were summarized in Table 1.

**Table 1:** Characteristics of the studies included in the meta-analysis.

Reference	Year	Ethnicity	Case	Control	No. of case	No. of control	Genotyping method
Cauchi [26]	2012	Arab	T2D per WHO criteria	Healthy	2639	1997	TaqMan
Cho [27]	2011	Asian	T2D patients	Non-diabetic participants	6952	11865	Genechip
Kooner [28]	2011	Asian	T2D patients	Non-diabetic participants	5561	14458	Genechip
Hu [29]	2010	Chinese	T2D per WHO criteria	Normal glucose tolerance	3410	3412	MassArray
Murad [30]	2010	British	T2D patients	Non-diabetic participants	1551	2993	TaqMan
Tam [31]	2010	Chinese	T2D per WHO criteria	Normal fasting glucose	1320	1595	MassArray
Dupuis [32]	2010	European, American, Austrian	T2D per WHO/ADA criteria	Non-diabetic participants	40655	87022	SNPstream, Genechip, TaqMan, MassArray
Ezzidi [33]	2009	Tunisian	T2D per ADA criteria	Normoglycemic participants	865	505	TaqMan
Prokopenko [18]	2009	European	T2D per WHO criteria; T2Dpatients	Normal glucose tolerant; Non-diabetic participants	11785	49799	Genechip
Reiling [34]	2009	Dutch	T2D per WHO criteria	Normal glucose tolerance	2498	1912	TaqMan
Qi [35]	2009	Chinese	T2D per WHO criteria	Normal fasting glucose	416	1877	SNPstream
Ma [36]	2009	Chinese	T2D per WHO criteria	Non-diabetic participants	279	110	RFLP
Cauchi [37]	2008	French	T2D per ADA criteria	Normoglycemic participants	2637	4159	TaqMan
Vaxillaire [12]	2008	French	T2D per ADA criteria	Normoglycemic participants	292	2752	TaqMan
Holmkvist [38]	2008	Swedish	T2D per ADA criteria	Non-diabetic participants	1988	15019	TaqMan
Winckler [39]	2007	British	T2D per WHO criteria	Non-diabetic participants	2248	3561	MassArray
Bonnycastle [40]	2006	Finnish	T2D per WHO criteria	Normal glucose tolerance	784	617	MassArray
Rose [14]	2005	Dane	T2D per WHO criteria	Normal glucose tolerance	1408	4773	MassArray
März [13]	2004	Austrian	T2D per ADA criteria	Non-diabetic participants	463	830	RFLP
Rissanen [41]	1998	Finnish	T2D patients	Normal glucose tolerance	36	294	SSCP
Yamada [16]	1997	Japanese	T2D per WHO criteria	Normal glucose tolerance	94	321	RFLP
Lotfi [42]	1997	Swedish	T2D per WHO criteria	Healthy	31	158	SSCP
Shimokawa [43]	1994	Japanese	T2D patients	Non-diabetic participants	240	111	SSCP
Chiu [44]	1994	American Blacks	T2D per NDDG criteria	Non-diabetic participants	77	99	SSCP

The article "Genetic Polymorphism of Glucokinase on the Risk of Type 2 Diabetes and Impaired Glucose Regulation: Evidence Based on 298, 468 Subjects" was retracted in 2021. Reasons: signs of a paper mill; concerns about the data; concerns about the authorship.

### Association of GCK −30G>A Variant with T2D

For T2D risk and the −30G>A polymorphism of *GCK*, our meta-analysis gave an overall OR of 1.06 (95% CI: 1.03–1.09; *P*<10^−4^; Fig. 1). Significantly increased T2D risks were also found under dominant (OR = 1.08; 95% CI: 1.01–1.19; *P* = 0.003) and recessive genetic models (OR = 1.12; 95% CI: 1.01–1.25; *P* = 0.008). This analysis is based on pooling of data from a number of different ethnic populations. When stratifying for ethnicity, an OR of 1.08 (95% CI: 1.04–1.12; *P*<10^−4^), 1.01 (95% CI: 0.98–1.05; *P* = 0.53) and 1.13 (95% CI: 1.04–1.24; *P* = 0.006) resulted for the A allele, among Caucasian, Asian and other ethnic population, respectively. Similar results were also detected using dominant and recessive genetic models (Table 2). When studies were stratified for sample size, significant risks were found among studies with small sample size in all genetic model (A allele: OR = 1.14, 95% CI: 1.04–1.25; dominant model: OR = 1.17, 95% CI: 1.06–1.28; recessive model: OR = 1.23, 95% CI: 1.05–1.43). Positive results still maintained for large sample size studies in all genetic models. Subsidiary analyses of diagnostic criterion yielded a per-allele OR for WHO criterion of 1.06 (95% CI: 1.01–1.11; *P* = 0.02), ADA criterion of 1.13 (95% CI: 0.99–1.28; *P* = 0.06) and for other criterion of 1.05 (95% CI: 0.99–1.11; *P* = 0.12).

**Figure 1:** Forest plot for the overall association between the *GCK*−30G>A polymorphism and type 2 diabetes risk.

**Table 2:** Meta-analysis of the *GCK* −30G>A polymorphism on type 2 diabetes risk.

Sub-group analysis	No. of data sets	No. of case/control	A allele				Dominant model				Recessive model			
			OR (95%CI)	P(Z)	P(Q)^a^	P(Q)^b^	OR (95%CI)	P(Z)	P(Q)^a^	P(Q)^b^	OR (95%CI)	P(Z)	P(Q)^a^	P(Q)^b^
Overall	36	88229/210239	1.06 (1.03–1.09)	<10^−4^	0.003		1.08 (1.01–1.19)	0.003	0.009		1.12 (1.01–1.25)	0.008	0.001	
Ethnicity						0.01				0.006				0.003
Caucasian	23	66376/173889	1.08 (1.04–1.12)	<10^−4^	0.002		1.13 (1.04–1.21)	0.0007	0.0006		1.17 (1.06–1.29)	0.002	<10^−4^	
Asian	9	18272/33749	1.01 (0.98–1.05)	0.53	0.77		0.96 (0.84–1.10)	0.57	0.82		1.05 (0.93–1.18)	0.76	0.34	
Others	4	3581/2601	1.13 (1.04–1.24)	0.006	0.49		1.06 (1.03–1.13)	0.008	0.63		1.12 (1.05–1.24)	0.03	0.52	
Sample size						0.001				0.006				<10^−4^
Small	15	4640/12804	1.14 (1.04–1.25)	0.006	0.09		1.17 (1.06–1.28)	0.009	0.21		1.23 (1.05–1.43)	0.01	0.10	
large	21	83589/197435	1.04 (1.01–1.07)	0.004	0.03		1.09 (1.02–1.23)	0.006	0.13		1.11 (1.07–1.35)	0.002	0.18	
Diagnostic criterion						0.44				0.53				0.14
WHO criterion	19	72385/169960	1.06 (1.01–1.11)	0.02	0.12		1.07 (1.02–1.19)	0.01	0.31		1.09 (1.05–1.17)	0.003	0.29	
ADA criterion	7	6247/23265	1.13 (0.99–1.28)	0.06	<10^−4^		1.06 (0.97–1.16)	0.13	<10^−4^		1.18 (0.94–1.47)	0.20	<10^−5^	
Other criterion	10	9597/17014	1.05 (0.99–1.11)	0.12	0.24		1.07 (0.97–1.19)	0.16	0.35		1.02 (0.87–1.19)	0.76	0.09	

a Cochran’s chi-square Q statistic test used to assess the heterogeneity in subgroups.

b Cochran’s chi-square Q statistic test used to assess the heterogeneity between subgroups.

The article "Genetic Polymorphism of Glucokinase on the Risk of Type 2 Diabetes and Impaired Glucose Regulation: Evidence Based on 298, 468 Subjects" was retracted in 2021. Reasons: signs of a paper mill; concerns about the data; concerns about the authorship.

Significant heterogeneity was present among the included studies (*P*<0.05). In meta-regression analysis, mean age of cases (*P* = 0.31) and controls (*P* = 0.24) and genotyping method (*P* = 0.96) did not significantly explain such heterogeneity. By contrast, ethnicity (*P* = 0.02) and the sample size in cases (*P* = 0.01) was significantly correlated with the magnitude of the genetic effect, explaining 11% and 16% of the heterogeneity, respectively. Since significant between-study heterogeneity still maintained in Caucasian subgroup, hence studies on Caucasian populations is the main source of heterogeneity.

### Association of GCK −30G>A Variant with Impaired Glucose Regulation

To investigate how glucose metabolism was related to glucokinase, we analyzed individuals with impaired glucose regulation (impaired glucose tolerance and/or impaired fasting glucose). The data on genotypes of the −30G>A polymorphism among impaired glucose regulation cases and controls were available in 5 (including 3177 cases and 8970 controls) studies. In the overall analysis, the −30G>A polymorphism of *GCK* was significantly associated with elevated impaired glucose regulation risk with a per-allele OR of 1.23 [95% CI: 1.14–1.32; *P*(Z) <10^−5^; *P*(Q) = 0.73; Fig. 2]. Significant associations were also found under dominant [OR = 1.24; 95% CI: 1.13–1.35; *P*(Z) <10^−5^; *P*(Q) = 0.56] and recessive [OR = 1.52; 95% CI: 1.20–1.91; *P*(Z) = 0.004; *P*(Q) = 0.77] genetic model.

The article "Genetic Polymorphism of Glucokinase on the Risk of Type 2 Diabetes and Impaired Glucose Regulation: Evidence Based on 298, 468 Subjects" was retracted in 2021. Reasons: signs of a paper mill; concerns about the data; concerns about the authorship.

**Figure 2:** Forest plot for the overall association between the *GCK*−30G>A polymorphism and impaired glucose regulation risk.

### Association of GCK −30G>A Variant with Fasting Plasma Glucose Level

The data on fasting plasma glucose (FPG) level among subjects stratified by genotype of −30G>A polymorphism were available in 6 studies, including 31,616 subjects. Significant increases of fasting plasma glucose level were observed in A allele carriers compared with non-carriers. Using the random-effects model, compared with G/G genotype, the WMD for heterozygous were 0.07 [95%: 0.05–0.08, *P(Z)* <10^−5^, *P(Q)* <10^−5^; Figure 3] and homozygous 0.15 [95%:0.05–0.24, *P(Z)* = 0.001, *P(Q)*<10^−5^], respectively.

**Figure 3:** Meta-analysis of weighted mean differences (WMD) of fasting plasma glucose levels between GG and GA genotype of −30G>A polymorphism.

### Sensitivity Analyses and Publication Bias

Sensitivity analysis indicated that no single study influenced the pooled OR qualitatively, suggesting that the results of this meta-analysis are stable (data not shown). The shape of the funnel plots was symmetrical (Figure S2). The statistical results still did not show publication bias in these studies (Begg test, P = 0.21; Egger test, *P* = 0.60).

## Discussion

Large sample and unbiased epidemiological studies of predisposition genes polymorphisms could provide insight into the in vivo relationship between candidate genes and diseases. This is the most comprehensive meta-analysis examining the *GCK* −30G>A polymorphism and the relationship to T2D risk. Its strength was based on the accumulation of published data giving greater information to detect significant differences. In total, the present meta-analysis combined 24 studies for T2D including 88, 229 cases and 210, 239 controls. Our results demonstrated that a modest association existed between the −30G>A variant of *GCK* and T2D risk.

In meta-analysis, heterogeneity evaluation was always conducted in statistical analysis. Thus, several subgroup meta-analyses were performed. In the stratified analysis by ethnicity, significant associations were found in Caucasians for the polymorphism in all genetic models; while no associations were detected among Asians. There are several possible reasons for such differences. First, the distribution of the A allele varies extensively between different races, with a prevalence of ∼23% among Asians and ∼17% among Caucasians. Therefore, additional studies are warranted to further validate ethnic difference in the effect of this polymorphism on T2D risk. In addition, different populations usually have different linkage disequilibrium patterns. A polymorphism may be in close linkage with another nearby causal variant in one ethnic population but not in another. *GCK* −30G>A polymorphism may be in close linkage with different nearby causal variants in different populations. Moreover, clinical heterogeneity like age, sex ratio, dietary, years from onset and disease severity may also explain the discrepancy. Finally, such different results could also be explained by study design or sample size. As significant between-study heterogeneity was found among Caucasian subgroup, so the result must be interpreted with caution since the Caucasian population reports in the subgroup analysis include a mixture of populations from very distant countries.

The article "Genetic Polymorphism of Glucokinase on the Risk of Type 2 Diabetes and Impaired Glucose Regulation: Evidence Based on 298, 468 Subjects" was retracted in 2021. Reasons: signs of a paper mill; concerns about the data; concerns about the authorship.

The present study also provides evidence that the −30G>A polymorphism of *GCK* influences susceptibility to phenotypes of impaired glucose regulation. In terms of genetic versus environmental influences on T2D susceptibility, this finding supports previous heritability studies, including a Danish twin study, generating considerably higher heritability estimates for the impaired glucose tolerance state compared with manifest T2D [42].

We also observed a significant effect of the −30G>A variant on FPG levels. This confirms a recent observation in a French study [12]. Therefore, this variant may have a non-negligible impact on human health. Indeed, there is strong evidence that even small changes in FPG, well below the impaired fasting glucose threshold of 6.1 mmol/l, may be associated with risk of cardiovascular morbidity and mortality [43], [44]. In this context, the *GCK* (−30A) allele was previously shown to be associated with type 2 diabetes and increased risk for coronary heart diseases in both diabetic and nondiabetic samples [13]. The exact mechanism by which the *GCK* −30A allele causes hyperglycemia is uncertain, but its effect seems constant throughout the lifespan, although insulin secretion is known to decrease with age in the general population. This is in accordance with the constant effect of the *GCK* −30A allele on fasting glucose reported in several groups of normoglycemic subjects whose median age varied from 8 to 72 years [12].

A number of factors predict T2D; however, detailed pathogenesis mechanisms of T2D remain a matter of speculation. GCK is a key regulatory enzyme in the pancreatic β-cell, and it plays a crucial role in determining the threshold for glucose-stimulated insulin secretion. Heterozygous inactivating mutations in GCK cause maturity-onset diabetes of the young subtype 2, in which hyperglycemia is present from birth. The decreased expression of functional GCK seems to be the cause of the observed hyperglycemia among maturity-onset diabetes of the young subtype 2 patients. The mechanism by which the −30G>A polymorphism causes hyperglycemia is uncertain. Previously studies suggested that the minor A allele or a genetic variant with which it is in linkage disequilibrium may alters the expression of *GCK* [14].

The article "Genetic Polymorphism of Glucokinase on the Risk of Type 2 Diabetes and Impaired Glucose Regulation: Evidence Based on 298, 468 Subjects" was retracted in 2021. Reasons: signs of a paper mill; concerns about the data; concerns about the authorship.

In interpreting the results, some limitations of this meta-analysis should be addressed. Firstly, in the subgroup analyses, different ethnicities were pooled in the other ethnic group which may bring in some heterogeneity. As studies among the other ethnic group are currently limited, further studies including a wider spectrum of subjects should be carried to investigate the role of these variants in different populations. Secondly, our results were based on unadjusted estimates, while a more precise analysis should be conducted if all individual raw data were available, which would allow for the adjustment by other co-variants including age, drinking status, obesity, cigarette consumption, and other lifestyle. Thirdly, only published studies were included in this meta-analysis. Therefore, publication bias may have occurred, even though the use of a statistical test did not show it.

Despite these limitations, this meta-analysis suggests that *GCK* −30G>A polymorphism was significantly associated with increased risk of T2D, particularly in Caucasian population. In addition, *GCK* –30A allele is a true risk factor for the development of impaired glucose regulation, having a significant impact on FPG level.

## Supporting Information

Figure S1 Study selection process.
(TIF)

Figure S2 Begg’s funnel plot of *GCK* −30G>A polymorphism and T2D risk.
(TIF)

Checklist S1 (DOC)

## References

[1] ZegginiE, ScottLJ, SaxenaR, VoightBF, MarchiniJL, et al (2008) Meta-analysis of genome-wide association data and large-scale replication identified additional susceptibility loci for type 2 diabetes. Nat Genet 40: 638–645.1837290310.1038/ng.120PMC2672416

[2] McCarthyMI (2010) Genomics, type 2 diabetes, and obesity. N Engl J Med 363: 2339–2350.2114253610.1056/NEJMra0906948

[3] VoightBF, ScottLJ, SteinthorsdottirV, MorrisAP, DinaC, et al (2010) Twelve type 2 diabetes susceptibility loci identified through large-scale association analysis. Nat Genet 42: 579–589.2058182710.1038/ng.609PMC3080658

[4] MatschinskyFM (1996) Banting lecture 1995. A lesson in metabolic regulation inspired by the glucokinase glucose sensor paradigm. Diabetes 45: 223–241.854986910.2337/diab.45.2.223

[5] FroguelP, ZoualiH, VionnetN, VelhoG, VaxillaireM, et al (1993) Familial hyperglycemia due to mutations in glucokinase. Definition of a subtype of diabetes mellitus. N Engl J Med 328: 697–702.843372910.1056/NEJM199303113281005

The article "Genetic Polymorphism of Glucokinase on the Risk of Type 2 Diabetes and Impaired Glucose Regulation: Evidence Based on 298, 468 Subjects" was retracted in 2021. Reasons: signs of a paper mill; concerns about the data; concerns about the authorship.

[6] GloynAL (2003) Glucokinase (GCK) mutations in hyper- and hypoglycemia: maturity-onset diabetes of the young, permanent neonatal diabetes, and hyperinsulinemia of infancy. Hum Mutat 22: 353–362.1451794610.1002/humu.10277

[7] NjølstadPR, SøvikO, Cuesta-MuñozA, BjørkhaugL, MassaO, et al (2001) Neonatal diabetes mellitus due to complete glucokinase deficiency. N Engl J Med 344: 1588–1592.1137201010.1056/NEJM200105243442104

[8] ChristesenHB, JacobsenBB, OdiliS, BuettgerC, Cuesta-MunozA, et al (2002) The second activating glucokinase mutation (A456V): implications for glucose homeostasis and diabetes therapy. Diabetes 51: 1240–1246.1191695110.2337/diabetes.51.4.1240

[9] Cuesta-MuñozAL, HuopioH, OtonkoskiT, Gomez-ZumaqueroJM, Näntö-SalonenK, et al (2004) Severe persistent hyperinsulinemic hypoglycemia due to a de novo glucokinase mutation. Diabetes 53: 2164–2168.1527740210.2337/diabetes.53.8.2164

[10] GlaserB, KesavanP, HeymanM, DavisE, CuestaA, et al (1998) Familial hyperinsulinism caused by an activating glucokinase mutation. N Engl J Med 338: 226–230.943532810.1056/NEJM199801223380404

[11] GloynAL, NoordamK, WillemsenMA, EllardS, LamWW, et al (2003) Insights into the biochemical and genetic basis of glucokinase activation from naturally occurring hypoglycemia mutations. Diabetes 52: 2433–2440.1294178610.2337/diabetes.52.9.2433

[12] VaxillaireM, VeslotJ, DinaC, ProençaC, CauchiS, et al (2008) Impact of common type 2 diabetes risk polymorphisms in the DESIR prospective study. Diabetes 57: 244–254.1797795810.2337/db07-0615

[13] MärzW, NauckM, HoffmannMM, NagelD, BoehmBO, et al (2004) G(−30)A polymorphism in the pancreatic promoter of the glucokinase gene associated with angiographic coronary artery disease and type 2 diabetes mellitus. Circulation 109: 2844–2849.1517302910.1161/01.CIR.0000129306.44085.C4

[14] RoseCS, EkJ, UrhammerSA, GlümerC, Borch-JohnsenK, et al (2005) A −30G>A polymorphism of the beta-cell-specific glucokinase promoter associates with hyperglycemia in the general population of whites. Diabetes 54: 3026–3031.1618640910.2337/diabetes.54.10.3026

[15] StoneLM, KahnSE, FujimotoWY, DeebSS, PorteDJr (1996) A variation at position –30 of the beta-cell glucokinase gene promoter is associated with reduced beta-cell function in middle-aged Japanese-American men. Diabetes 45: 422–428.860376210.2337/diab.45.4.422

[16] YamadaK, YuanX, IshiyamaS, IchikawaF, KoyamaKI, et al (1997) Clinical characteristics of Japanese men with glucokinase gene beta-cell promoter variant. Diabetes Care 20: 1159–1161.920345510.2337/diacare.20.7.1159

The article "Genetic Polymorphism of Glucokinase on the Risk of Type 2 Diabetes and Impaired Glucose Regulation: Evidence Based on 298, 468 Subjects" was retracted in 2021. Reasons: signs of a paper mill; concerns about the data; concerns about the authorship.

[17] WeedonMN, ClarkVJ, QianY, Ben-ShlomoY, TimpsonN, et al (2006) A common haplotype of the glucokinase gene alters fasting glucose and birth weight: association in six studies and population-genetics analyses. Am J Hum Genet 79: 991–1001.1718645810.1086/509517PMC1698701

[18] ProkopenkoI, LangenbergC, FlorezJC, SaxenaR, SoranzoN, et al (2009) Variants in MTNR1B influence fasting glucose levels. Nat Genet 41: 77–81.1906090710.1038/ng.290PMC2682768

[19] CochranWG (1954) The combination of estimates from different experiments. Biometrics 10: 101–129.

[20] DerSimonianR, LairdN (1896) Meta-analysis in clinical trials. Control Clin Trial 7: 177–188.10.1016/0197-2456(86)90046-23802833

[21] ThompsonSG, SharpSJ (1999) Explaining heterogeneity in meta-analysis: a comparison of methods. Stat Med 18: 2693–2708.1052186010.1002/(sici)1097-0258(19991030)18:20<2693::aid-sim235>3.0.co;2-v

[22] EggerM, Davey SmithG, SchneiderM, MinderC (1997) Bias in meta-analysis detected by a simple, graphical test. BMJ 315: 629–634.931056310.1136/bmj.315.7109.629PMC2127453

[23] CauchiS, EzzidiI, El AchhabY, MtiraouiN, ChaiebL, et al (2012) European genetic variants associated with type 2 diabetes in North African Arabs. Diabetes Metab 38: 316–323.2246397410.1016/j.diabet.2012.02.003

[24] ChoYS, ChenCH, HuC, LongJ, OngRT, et al (2011) Meta-analysis of genome-wide association studies identifies eight new loci for type 2 diabetes in east Asians. Nat Genet 44: 67–72.2215853710.1038/ng.1019PMC3582398

[25] KoonerJS, SaleheenD, SimX, SehmiJ, ZhangW, et al (2011) Genome-wide association study in individuals of South Asian ancestry identifies six new type 2 diabetes susceptibility loci. Nat Genet 43: 984–989.2187400110.1038/ng.921PMC3773920

[26] HuC, ZhangR, WangC, YuW, LuJ, et al (2010) Effects of GCK, GCKR, G6PC2 and MTNR1B variants on glucose metabolism and insulin secretion. PloS One 5: e11761.2066870010.1371/journal.pone.0011761PMC2909258

[27] MuradAS, SmithGD, LewisSJ, CoxA, DonovanJL, et al (2010) A polymorphism in the glucokinase gene that raises plasma fasting glucose, rs1799884, is associated with diabetes mellitus and prostate cancer: findings from a population-based, case-control study (the ProtecT study). Int J Mol Epidemiol Genet 1: 175–183.21537389PMC3076770

[28] TamCH, HoJS, WangY, LeeHM, LamVK, et al (2010) Common polymorphisms in MTNR1B, G6PC2 and GCK are associated with increased fasting plasma glucose and impaired beta-cell function in Chinese subjects. PloS One 5: e11428.2062859810.1371/journal.pone.0011428PMC2900202

[29] DupuisJ, LangenbergC, ProkopenkoI, SaxenaR, SoranzoN, et al (2010) New genetic loci implicated in fasting glucose homeostasis and their impact on type 2 diabetes risk. Nat Genet 42: 105–116.2008185810.1038/ng.520PMC3018764

The article "Genetic Polymorphism of Glucokinase on the Risk of Type 2 Diabetes and Impaired Glucose Regulation: Evidence Based on 298, 468 Subjects" was retracted in 2021. Reasons: signs of a paper mill; concerns about the data; concerns about the authorship.

[30] EzzidiI, MtiraouiN, CauchiS, VaillantE, DechaumeA, et al (2009) Contribution of type 2 diabetes associated loci in the Arabic population from Tunisia: a case-control study. BMC Med Genet 10: 33.1936870710.1186/1471-2350-10-33PMC2678106

[31] ReilingE, van ‘t RietE, GroenewoudMJ, WelschenLM, van HoveEC, et al (2009) Combined effects of single-nucleotide polymorphisms in GCK, GCKR, G6PC2 and MTNR1B on fasting plasma glucose and type 2 diabetes risk. Diabetologia 52: 1866–1870.1953308410.1007/s00125-009-1413-9PMC2723681

[32] QiQ, WuY, LiH, LoosRJ, HuFB, et al (2009) Association of GCKR rs780094, alone or in combination with GCK rs1799884, with type 2 diabetes and related traits in a Han Chinese population. Diabetologia 52: 834–843.1924105810.1007/s00125-009-1290-2

[33] MaYC, WangYM (2009) Study of the correlation between the variation at −30 position of glucokinase gene promoter and type 2 diabetes. Zhongguo xian dai yi xue yuan zha zhi 19: 513–520.

[34] CauchiS, NeadKT, ChoquetH, HorberF, PotocznaN, et al (2008) The genetic susceptibility to type 2 diabetes may be modulated by obesity status: implications for association studies. BMC Med Genet 9: 45.1849863410.1186/1471-2350-9-45PMC2412856

[35] HolmkvistJ, AlmgrenP, LyssenkoV, LindgrenCM, ErikssonKF, et al (2008) Common variants in maturity-onset diabetes of the young genes and future risk of type 2 diabetes. Diabetes 57: 1738–1744.1833210110.2337/db06-1464

[36] WincklerW, WeedonMN, GrahamRR, McCarrollSA, PurcellS, et al (2007) Evaluation of common variants in the six known maturity-onset diabetes of the young (MODY) genes for association with type 2 diabetes. Diabetes 56: 685–693.1732743610.2337/db06-0202

[37] BonnycastleLL, WillerCJ, ConneelyKN, JacksonAU, BurrillCP, et al (2006) Common variants in maturity-onset diabetes of the young genes contribute to risk of type 2 diabetes in Finns. Diabetes 55: 2534–2540.1693620110.2337/db06-0178

[38] RissanenJ, SaarinenL, HeikkinenS, KekäläinenP, MykkänenL, et al (1998) Glucokinase gene islet promoter region variant (GA) at nucleotide −30 is not associated with reduced insulin secretion in Finns. Diabetes Care 21: 1194–1197.965361910.2337/diacare.21.7.1194

[39] LotfiK, SundG, LoweR, GrahamJ, Landin-OlssonM, et al (1997) The beta cell glucokinase promoter variant is an unlikely risk factor for diabetes mellitus. Diabetes Incidence Study in Sweden (DISS). Diabetologia 40: 959–962.926799210.1007/s001250050774

[40] ShimokawaK, SakuraH, OtabeS, EtoK, KadowakiH, et al (1994) Analysis of the glucokinase gene promoter in Japanese subjects with noninsulin-dependent diabetes mellitus. J Clin Endocrinol Metab 79: 883–886.807737610.1210/jcem.79.3.8077376

The article "Genetic Polymorphism of Glucokinase on the Risk of Type 2 Diabetes and Impaired Glucose Regulation: Evidence Based on 298, 468 Subjects" was retracted in 2021. Reasons: signs of a paper mill; concerns about the data; concerns about the authorship.

[41] ChiuKC, GoRC, AokiM, RiggsAC, TanizawaY, et al (1994) Glucokinase gene in gestational diabetes mellitus: population association study and molecular scanning. Diabetologia 37: 104–110.815022210.1007/BF00428785

[42] PoulsenP, KyvikKO, VaagA, Beck-NielsenH (1999) Heritability of type II (non-insulin-dependent) diabetes mellitus and abnormal glucose tolerance: a population-based twin study. Diabetologia 42: 139–145.1006409210.1007/s001250051131

[43] CoutinhoM, GersteinHC, WangY, YusufS (1999) The relationship between glucose and incident cardiovascular events: a metaregression analysis of published data from 20 studies of 95,783 individuals followed for 12.4 years. Diabetes Care 22: 233–240.1033393910.2337/diacare.22.2.233

[44] PanzerC, LauerMS, BriekeA, BlackstoneE, HoogwerfB (2002) Association of fasting plasma glucose with heart rate recovery in healthy adults: a population-based study. Diabetes 51: 803–807.1187268310.2337/diabetes.51.3.803

